# Open Resection Compared to Mini-Invasive in Colorectal Cancer and Liver Metastases: A Meta-Analysis

**DOI:** 10.3389/fsurg.2021.726217

**Published:** 2021-08-30

**Authors:** Jie Gong, Fengwei Gao, Qingyun Xie, Xin Zhao, Zehua Lei

**Affiliations:** Department of Hepatobiliary and Pancreatic Spleen, Leshan People's Hospital, Leshan, China

**Keywords:** minimally invasive surgery, colorectal cancer, synchronous colorectal liver metastases, open surgery, operation time, preoperative complication, postoperative complication

## Abstract

**Background:** We performed a meta-analysis to evaluate the outcomes of minimally invasive surgery and open surgery in the simultaneous resection of colorectal cancer and synchronous colorectal liver metastases.

**Methods:** A systematic literature search up to April 2021 was done and 13 studies included 1,181 subjects with colorectal cancer and synchronous colorectal liver metastases at the start of the study; 425 of them were using minimally invasive surgery and 756 were open surgery. They were reporting relationships between the outcomes of minimally invasive surgery and open surgery in the simultaneous resection of colorectal cancer and synchronous colorectal liver metastases. We calculated the odds ratio (OR) or the mean difference (MD) with 95% CIs to assess the outcomes of minimally invasive surgery and open surgery in the simultaneous resection of colorectal cancer and synchronous colorectal liver metastases using the dichotomous or continuous method with a random or fixed-effect model.

**Results:** Minimally invasive surgery in subjects with colorectal cancer and synchronous colorectal liver metastases was significantly related to longer operation time (MD, 35.61; 95% CI, 7.36–63.87, *p* = 0.01), less blood loss (MD, −151.62; 95% CI, −228.84 to −74.40, *p* < 0.001), less blood transfusion needs (OR, 0.61; 95% CI, 0.42–0.89, *p* = 0.01), shorter length of hospital stay (MD, −3.26; 95% CI, −3.67 to −2.86, *p* < 0.001), lower overall complications (OR, 0.59; 95% CI, 0.45–0.79, *p* < 0.001), higher overall survival (OR, 1.66; 95% CI, 1.21–2.29, *p* = 0.002), and higher disease-free survival (OR, 1.49; 95% CI, 1.13–1.97, *p* = 0.005) compared to open surgery.

**Conclusions:** Minimally invasive surgery in subjects with colorectal cancer and synchronous colorectal liver metastases may have less blood loss, less blood transfusion needs, shorter length of hospital stay, lower overall complications, higher overall survival, and higher disease-free survival with longer operation time compared with the open surgery. Furthers studies are required to validate these findings.

## Background

Colorectal cancer is one of the main reasons for cancer-related mortality in the world. The frequency and death of colorectal cancer are the third and the second, respectively, of all types of cancer in the world (1). According to the last global cancer report by the International Agency for Research on Cancer for 2018, more than 1,800,000 subjects were newly diagnosed with colorectal cancer, and about one million subjects died from colorectal cancer (1). The liver is the common organ for metastasis from colorectal cancer. Almost 40% of subjects with colorectal cancer progress to liver metastases, and 15–20% of colorectal cancer subjects have synchronous colorectal liver metastases at the time of diagnosis; the metastases are restricted to the liver in 70–80% of those subjects, but a limited subset of these metastases are resectable (2). Radical resection of primary and metastatic lesions is a possible curative treatment strategy for subjects with resectable colorectal cancer and synchronous colorectal liver metastases (3). The resection techniques for colorectal cancer and synchronous colorectal liver metastases are simultaneous resection and staged resection. Staged resection of the initial tumor and synchronous colorectal liver metastases was first done by removing the primary colorectal cancer tumor, followed by adjuvant chemotherapy and liver metastasis tumor resection (4). Lately, several studies have recommended that the simultaneous resection of primary colorectal cancer and synchronous colorectal liver metastases. They suggested that this technique is acceptable, safe, and may turn into an optimum management strategy for subjects with resectable colorectal cancer and synchronous colorectal liver metastases (5, 6). Simultaneous resection of colorectal cancer and synchronous colorectal liver metastases was only done by open surgery before minimally invasive surgery e.g., laparoscopy or robotics was applied in the management of colorectal cancer (7). Minimally invasive surgery showed better short-term and similar long-term management results to conventional open surgery in some studies (8–10). Though, most of the studies were case series or case reports with small sample sizes (11, 12). The benefits of minimally invasive surgery over open surgery are still unclear, mainly the long-term results. So, this meta-analysis was performed to evaluate the outcomes of minimally invasive surgery and open surgery in the simultaneous resection of colorectal cancer and synchronous colorectal liver metastases.

## Methods

The present study followed the meta-analysis of studies in the epidemiology statement (13), which was performed following an established protocol.

### Study Selection

Included studies were that with statistical measures of relationship (odds ratio [OR], mean difference [MD], frequency rate ratio, or relative risk, with 95% CI) between the outcomes of minimally invasive surgery and open surgery in the simultaneous resection of colorectal cancer and synchronous colorectal liver metastases.

Only human studies in any language were considered. Inclusion was not restricted by study size or type. Publications excluded were review articles and commentary and studies that did not supply a degree of relationship. Figure 1 shows the whole study process.

**Figure 1:** Schematic diagram of the study procedure.

The articles were included in the meta-analysis when the next inclusion criteria were met:

1. The study was a randomized control trial or retrospective study.
2. The target population is subjects with colorectal cancer and synchronous colorectal liver metastases.
3. The intervention program was the minimally invasive surgery and open surgery.
4. The study included comparisons between the outcomes of minimally invasive surgery and open surgery in the simultaneous resection of colorectal cancer and synchronous colorectal liver metastases.

The exclusion criteria were as follows:

1. Studies that did not compare minimally invasive surgery to open surgery.
2. Studies with diseases other than colorectal cancer and synchronous colorectal liver metastases.
3. Studies did not focus on the effect on comparative results.

### Identification

A protocol of search strategies was prepared according to the PICOS principle (14), and we defined it as follow: P (population): subjects with colorectal cancer and synchronous colorectal liver metastases; I (intervention/exposure): minimally invasive surgery and open surgery; C (comparison): outcomes of minimally invasive surgery and open surgery in the simultaneous resection of colorectal cancer and synchronous colorectal liver metastases; O (outcome): operation time, preoperative, and postoperative complications; and S (study design): no restriction (15). First, we conducted a systematic search of Embase, PubMed, Cochrane Library, OVID, and Google scholar till April 2021, by a blend of keywords and related words for minimally invasive surgery, colorectal cancer, synchronous colorectal liver metastases, open surgery, operation time, preoperative complication, and postoperative complication as shown in Table 1. All selected studies were gathered in an EndNote file, duplicates were removed, and the title and abstracts were revised to eliminate studies that did not report a relationship between the outcomes of minimally invasive surgery and open surgery in the simultaneous resection of colorectal cancer and synchronous colorectal liver metastases. The remaining articles were revised for related information.

**Table 1:** Search strategy for each database.

**Database**	**Search strategy**
Pubmed	#1 “minimally invasive surgery” [MeSH Terms] OR “colorectal cancer” [All Fields] OR “synchronous colorectal liver metastases” [All Fields] OR “open surgery” [All Fields]
	#2 “operation time” [MeSH Terms] OR “minimally invasive surgery” [All Fields] OR “Preoperative complication” [All Fields] OR “postoperative complication” [All Fields]
	#3 #1 AND #2
Embase	‘minimally invasive surgery'/exp OR ‘colorectal cancer'/exp OR ‘synchronous colorectal liver metastases'/exp OR ‘open surgery'/exp
	#2 ‘operation time'/exp OR ‘ICBG'/exp OR ‘Preoperative complication'/exp OR ‘postoperative complication'/exp
	#3 #1 AND #2
Cochrane library	#1 (minimally invasive surgery):ti,ab,kw OR (colorectal cancer):ti,ab,kw OR (synchronous colorectal liver metastases):ti,ab,kw OR (open surgery):ti,ab,kw (Word variations have been searched)
	#2 (operation time):ti,ab,kw OR (Preoperative complication):ti,ab,kw OR (postoperative complication):ti,ab,kw (Word variations have been searched)
	#3 #1 AND #2

### Screening

Data were abbreviated based on the following; study associated and subject associated features onto a homogeneous form, the primary author last name, study period, publication year, country, the studies region, and design of the study; type of the population, the total number and subjects number, demographic data and clinical and treatment features; the evaluation period associated to measurement, quantitative method and qualitative method of assessment, source of information, and assessment of the outcomes; and statistical analysis MD or relative risk, with 95% CI of relationship among the outcomes of minimally invasive surgery and open surgery in the simultaneous resection of colorectal cancer and synchronous colorectal liver metastases (16). If a study fit for inclusion based upon the abovementioned principles, data were extracted individually by two authors. In case of discrepancy, the corresponding author gave a final choice. When there were diverse data from a study, the data were extracted separately. The bias risk in the studies; each study was assessed using two authors who individually evaluated the methodological quality of the selected studies. We used the “risk of bias tool” from the RoB 2: a revised Cochrane risk-of-bias tool for randomized trials to evaluate methodological quality (17). In terms of the evaluation criteria, each study was valued and allocated to one of the next three risks of bias: low: if all quality criteria were met; unclear or moderate: if one or more of the quality criteria were partly met or unclear, or high: if one or more of the criteria were not met, or not included. Any discrepancies were addressed by a reassessment of the original article.

### Eligibility

The main result concentrated on measuring minimally invasive surgery and open surgery in the simultaneous resection of colorectal cancer and synchronous colorectal liver metastases. An assessment of the outcomes of minimally invasive surgery and open surgery in the simultaneous resection of colorectal cancer and synchronous colorectal liver metastases was extracted forming a summary.

### Inclusion

Sensitivity analyses were limited only to studies reporting the relationship between the outcomes of minimally invasive surgery and open surgery in the simultaneous resection of colorectal cancer and synchronous colorectal liver metastases. For subcategory and sensitivity analysis, we compared the effect of minimally invasive surgery to open surgery.

### Statistical Analysis

The dichotomous or continuous method with random-effect or fixed-effect models was used to calculate the OR or MD and 95% CI. We used the Chi-square test to perform biological heterogeneity analyses between different studies. We calculated the *I*^2^ index; the *I*^2^ index is from 0 to 100%. Values of about 0, 25, 50, and 75% indicate no, low, moderate, and high heterogeneity, respectively (18). When *I*^2^ was higher than 50%, we chose the random effect model; when it was lower than 50%, we used the fixed-effect model. A subgroup analysis was performed by stratifying the original evaluation per liver cancer and chemotherapy different outcomes as described before. In this analysis, a *p*-value for differences between subgroups of <0.05 was considered statistically significant. Publication bias was evaluated quantitatively using the Egger regression test (publication bias considered present if *p* ≥ 0.05), and qualitatively, by visual examination of funnel plots of the logarithm of ORs or MDs vs. their SE (16). All *p*-values were 2 tailed. All calculations and graphs were performed using Reviewer manager version 5.3 (The Nordic Cochrane Center, The Cochrane Collaboration, Copenhagen, Denmark).

## Results

A total of 2,534 unique studies were identified, of which 13 studies (between 2011 and 2021) fulfilled the inclusion criteria and were included in the study (19–31).

The 13 studies included 1,181 subjects with colorectal cancer and synchronous colorectal liver metastases at the start of the study; 425 of them were using minimally invasive surgery and 756 were open surgery. All studies evaluated the outcomes of minimally invasive surgery and open surgery in the simultaneous resection of colorectal cancer and synchronous colorectal liver metastases.

Study size ranged from 14 to 444 subjects with colorectal cancer and synchronous colorectal liver metastases at the start of the study. The details of the 13 studies are shown in Table 2. Thirteen studies reported data stratified to operation time, 12 studies stratified to the blood loss, 10 studies reported data stratified to studies stratified to blood transfusion needs, 12 studies reported data stratified to the length of hospital stay, 12 studies stratified to the overall complications, nine studies stratified to the overall survival, and nine studies stratified to disease-free survival.

**Table 2:** Characteristics of the selected studies for the meta-analysis.

**Study**	**Country**	**Total**	**Minimally invasive surgery**	**Open surgery**
Chen et al. (19)	China	41	23	18
Hu et al. (20)	China	26	13	13
Takasu et al. (21)	Japan	14	7	7
Lin et al. (22)	China	72	36	36
Ratti et al. (23)	Italy	75	25	50
Tranchart et al. (24)	France	178	89	89
Gorgun et al. (25)	USA	43	14	29
Ivanecz et al. (26)	Slovenia	20	10	10
Chen et al. (27)	Taiwan	38	16	22
Shin et al. (28)	South Korea	444	126	318
Taesombat et al. (29)	Thailand	36	12	24
Nozawa et al. (30)	Japan	53	17	36
Kawakatsu et al. (31)	Japan	141	37	104
	**Total**	**1,181**	**425**	**756**

Minimally invasive surgery in subjects with colorectal cancer and synchronous colorectal liver metastases was significantly related to longer operation time (MD, 35.61; 95% CI, 7.36–63.87, *p* = 0. 01) with high heterogeneity (*I*^2^ = 84%), less blood loss (MD, −151.62; 95% CI, −228.84 to −74.40, *p* < 0.001) with high heterogeneity (*I*^2^ = 90%), less blood transfusion needs (OR, 0.61; 95% CI, 0.42–0.89, *p* = 0.01) with no heterogeneity (*I*^2^ = 0%), shorter length of hospital stay (MD, −3.26; 95% CI, −3.67 to−2.86, *p* < 0.001) with low heterogeneity (*I*^2^ = 41%), lower overall complications (OR, 0.59; 95% CI, 0.45–79, *p* < 0.001) with no heterogeneity (*I*^2^ = 0%), higher overall survival (OR, 1.66; 95% CI, 1.21–2.29, *p* = 0.002) with no heterogeneity (*I*^2^ = 0%), and higher disease-free survival (OR, 1.49; 95% CI, 1.13–1.97, *p* = 0.005) with no heterogeneity (*I*^2^ = 0%) compared to open surgery as shown in Figures 2–8.

**Figure 2:** Forest plot of the effect of minimally invasive surgery compared to open surgery on operation time in subjects with colorectal cancer and synchronous colorectal liver metastases.

**Figure 3:** Forest plot of the effect of minimally invasive surgery compared to open surgery on the blood loss in subjects with colorectal cancer and synchronous colorectal liver metastases.

**Figure 4:** Forest plot of the effect of minimally invasive surgery compared to open surgery on blood transfusion needs in subjects with colorectal cancer and synchronous colorectal liver metastases.

**Figure 5:** Forest plot of the effect of minimally invasive surgery compared to open surgery on the length of hospital stay in subjects with colorectal cancer and synchronous colorectal liver metastases.

**Figure 6:** Forest plot of the effect of minimally invasive surgery compared to open surgery on overall complications in subjects with colorectal cancer and synchronous colorectal liver metastases.

**Figure 7:** Forest plot of the effect of minimally invasive surgery compared to open surgery on overall survival in subjects with colorectal cancer and synchronous colorectal liver metastases.

**Figure 8:** Forest plot of the effect of minimally invasive surgery compared to open surgery on disease-free survival in subjects with colorectal cancer and synchronous colorectal liver metastases.

Selected studies stratified analysis that did and did not adjust for age, and ethnicity was not performed since no studies reported or adjusted for these factors.

Based on the visual examination of the funnel plot and on quantitative measurement by the Egger regression test, there was no indication of publication bias (*p* = 0.85). Though, most of the comprised studies were evaluated to be of a low methodological quality. All studies did not have selective reporting bias, and no articles had incomplete result data and selective reporting.

## Discussion

This meta-analysis study based on 13 studies included 1,181 subjects with colorectal cancer and synchronous colorectal liver metastases at the start of the study; 425 of them were using minimally invasive surgery and 756 were open surgery (19–31). Minimally invasive surgery in subjects with colorectal cancer and synchronous colorectal liver metastases was significantly related to longer operation time, less blood loss, less blood transfusion needs, shorter length of hospital stay, lower overall complications, higher overall survival, and higher disease-free survival compared to open surgery (19–31). Though, the analysis of outcomes should be done with caution because of the low sample size of most of the selected studies (10 studies were ≤ 100 subjects) in the meta-analysis especially in some parameters; suggesting the need for more studies comparing minimally invasive surgery to open surgery in subjects with colorectal cancer and synchronous colorectal liver metastases to validate these findings or possibly to significantly influence confidence in the effect evaluation.

The resection timing of primary colorectal cancer and synchronous colorectal liver metastases has been well studied. Some Studies suggested that staged resection decreases the preoperative and postoperative complications and makes the occult micrometastases perceptible (32, 33). Though, some others believe that simultaneous resection can decrease the tumor burden and economic and psychological burden of the subjects, making the subjects experiencing one operation instead of two (4, 34). Lately, with the advances in perioperative management and critical care, the operation timing for resectable subjects progressively changed from staged resection to simultaneous resection (35–37). Simultaneous resection of primary colorectal cancer and synchronous colorectal liver metastases is frequently done by open surgery. In open surgery surgeon always needs a long abdominal incision for satisfactory exposure of the operative field, leading to severe pain and incision complications (20). Open surgery is also related to serious physical and psychological operation trauma to the subjects. That may increase blood loss, the blood transfusion needs, and the length of hospital stay of the subject under open surgery as shown in the results (8–10). With the developments in surgical methods and tools, minimally invasive surgery showed some advantages in some surgeries such as proctocolectomy or hepatectomy (7, 8). Though, the results showed that the minimally invasive surgery had a significantly longer operation time compared to open surgery. That could be because the operation time depended on the features of primary tumors and liver metastases, the experience of the surgical teams, and the severe degree of abdominal adhesion and obesity (38, 39). These parameters could extend operation time in minimally invasive surgery compared to open surgery (38, 39). The safety of the minimally invasive surgery was proved here to be better than that of open surgery as shown in the significant difference found between minimally invasive surgery and open surgery in overall complications, overall survival, and disease-free survival (8–10).

This meta-analysis showed the relationship between minimally invasive surgery effects in subjects with colorectal cancer and synchronous colorectal liver metastases compared to open surgery. However, further studies are needed to validate these potential relationships. Also, further studies are needed to deliver a clinically meaningful difference in the results. These studies must comprise larger with more homogeneous samples. This was also suggested before in a similar meta-analysis study that showed a similar effect of minimally invasive surgery and open surgery in subjects with colorectal cancer and synchronous colorectal liver metastases (9, 10, 40). Well-conducted studies are also required to evaluate these factors and the combination of different subject-level data, age, and ethnicity; since our meta-analysis study could not answer whether they are related to the outcomes. In summary, the data suggest that minimally invasive surgery in subjects with colorectal cancer and synchronous colorectal liver metastases may have less blood loss, less blood transfusion needs, shorter length of hospital stay, lower overall complications, higher overall survival, and higher disease-free survival with longer operation time compared to open surgery. Furthers studies are required to validate these findings.

### Limitations

There may be selection bias in this study because many studies selected were excluded from the meta-analysis. Though, the excluded studies did not fulfill the inclusion criteria of the meta-analysis. Also, whether the results are associated with age and ethnicity or not could not be answered. The study designed to evaluate the relationship between the outcomes of minimally invasive surgery and open surgery in the simultaneous resection of colorectal cancer and synchronous colorectal liver metastases was based on data from previous studies, which might cause bias induced by incomplete details. The meta-analysis was based on 13 studies; 10 studies were small, ≤ 100. Variables, namely, age, ethnicity, and nutritional status of subjects were also the possible bias-inducing factors. Some unpublished articles and missing data might lead to a bias in the pooled effect. Subjects were using different treatment schedules, dosages, and health care systems. Also, the surgeries were done by different surgical teams with different experiences and skills, different perioperative management, and different types of surgeries due to different tumor locations.

## Conclusions

Minimally invasive surgery in subjects with colorectal cancer and synchronous colorectal liver metastases may have a lower risk of blood loss, less blood transfusion needs, shorter length of hospital stay, lower overall complications, higher overall survival, and higher disease-free survival with longer operation time compared to open surgery.

Though, the analysis of outcomes should be done with caution because of the low sample size of most of the selected studies in the meta-analysis especially in some parameters; suggesting the need for more studies comparing minimally invasive surgery to open surgery in subjects with colorectal cancer and synchronous colorectal liver metastases to validate these findings. Additionally, the major limitation of our study was that we could not describe in more detail the type of liver surgery performed in both groups (open and minimally invasive) and the type of associated colorectal surgery since no enough data in the 13 selected papers described these parameters in more details. It is very relevant to know if the type of liver surgery performed was local resections or major hepatectomies (three or more liver segments). It seems essential to describe the type of liver and colorectal resections and whether or not there are significant differences with respect to major or minor hepatectomies in both branches. Hence, this suggests the further description of such parameters in the upcoming studies with more details.

## Data Availability Statement

The original contributions presented in the study are included in the article/supplementary material, further inquiries can be directed to the corresponding author/s.

## Author Contributions

JG: administrative support, provision of study materials or subjects, and manuscript writing. FG: administrative support, collection and assembly of data, and manuscript writing. QX: provision of study materials or subjects, data analysis, and interpretation. XZ: collection and assembly of data, data analysis and interpretation, and manuscript writing. ZL: conception and design, and final approval of the manuscript. All authors have read and approved the manuscript.

## Conflict of Interest

The authors declare that the research was conducted in the absence of any commercial or financial relationships that could be construed as a potential conflict of interest.

## Publisher's Note

All claims expressed in this article are solely those of the authors and do not necessarily represent those of their affiliated organizations, or those of the publisher, the editors and the reviewers. Any product that may be evaluated in this article, or claim that may be made by its manufacturer, is not guaranteed or endorsed by the publisher.

## Abbreviations

OR: odds ratio
CIs: confidence intervals.
